# Study on the Correlation between the Levels of HtrA3 and TGF-*β*2 in Late Pregnancy and Preeclampsia

**DOI:** 10.1155/2022/4453646

**Published:** 2022-01-07

**Authors:** Wenying Huang, Shuxuan Zhang

**Affiliations:** ^1^Xuzhou Medical University, Xuzhou 221000, Jiangsu, China; ^2^Department of Obstetrics, Tengzhou Maternity and Child Health Hospital, Tengzhou 277500, Shandong, China; ^3^Department of Obstetrics, Xuzhou First People's Hospital Affiliated to Xuzhou Medical University, Xuzhou 221004, Jiangsu, China

## Abstract

Preeclampsia (PE) is a common and proprietary complication during pregnancy. The correlation was found between the levels of HtrA3 and TGF-*β* 2 and preeclampsia (PE). This study aimed to detect the HtrA3 and TGF-*β*2 in different parts of the third trimester (maternal serum, placenta). The 102 pregnant women who were eligible for enrollment in the obstetric examination at Tengzhou Maternity and Child Health Hospital from June 2020 to December 2020 were selected as the research objects. 28 cases diagnosed with PE were set up as the observation group 1, and 24 cases diagnosed with severe PE were set up as the observation group 2. Select 50 normal pregnant women as the control group and research the expressions of HtrA3 and TGF-*β*2 in maternal blood and placental tissues of patients with PE. ELISA was used to measure the concentration of HtrA3 and TGF-*β*2 in maternal blood. The distribution of HtrA3 and TGF-*β*2 in the placenta was observed by immunohistochemical techniques (IHC) and mean optical density value (MOD). S/D was measured by using color Doppler ultrasonic. The concentration of HtrA3 and TGF-*β*2 in the maternal blood and placenta tissue was higher in severe PE compared with PE and normotensive pregnancy, respectively (*P* < 0.05). There is a negative correlation between the level of HtrA3 and TGF-*β*2 and the birthweight of newborns both in maternal plasma and placenta tissue in preeclampsia and positive correlation between HtrA3 and TGF-*β*2 levels and S/D. HtrA3 and TGF-*β*2 may correlate with severity of PE and their neonatal adverse outcomes.

## 1. Introduction

Preeclampsia (PE) refers to new hypertension, proteinuria, or multiple organ damage that cannot be explained by other diseases after 20 weeks of pregnancy. Severe cases can affect the safety of mothers and children, and the world's total incidence is 2–8% [1]. Nowadays, the pathogenesis has not been studied clearly, but most experts believe that one of the reasons for the onset of preeclampsia is insufficient trophoblast invasion [2]. HtrA3 is a widely distributed secreted protein and a member of the HtrA family. When trophoblast cells are planted and enter the myometrium to promote the formation of the placenta, HtrA3 can inhibit this process by regulating TGF-*β* signaling and has a certain relationship with the pathogenesis of preeclampsia. At present, the research on HtrA3 and preeclampsia mainly focuses on the early and second trimesters. Whether the expression of HtrA3 in various detection methods in the third trimester is related to preeclampsia and neonatal outcomes has not been reported yet. TGF-*β* can participate in the regulation of the severity of preeclampsia by influencing the transformation of the endometrium to decidua, controlling the penetration of trophoblasts into the myometrium, and inhibiting the formation of placenta. Its family mainly includes three groups of cytokines: TGF-*β*1, TGF-*β*2, and TGF-*β*3. Previous reports on TGF-*β*1 and TGF-*β*3 are more common, but there are few studies on the relationship between TGF-*β*2 and preeclampsia. The lower the ROD value of TGF-*β*2 mRNA and protein content, the greater the probability of preeclampsia and the more serious it is. It is speculated that the low expression of TGF-*β*2 is related to the condition and severity of the disease [3]. Yang et al. have different findings. Compared with the normal control group, the mRNA and protein content of placenta TGF-*β*2 and its receptor TGFRII in the preeclampsia group were significantly higher [3, 4]. The results of this experiment show that the expression level of TGF-*β*2 in the maternal serum and placenta tissue of patients with preeclampsia is higher than that of normal placenta, which is contrary to the results of Zejun et al. but is consistent with the results of Xiuhua et al. The above experiments and discussion have confirmed that TGF-*β*2 has a certain correlation with the occurrence of preeclampsia.

The purpose of this study was to detect HtrA3 and TGF-*β*2 in different parts of the third trimester (maternal serum, placenta) in order to further explore the correlation between the expression levels of HtrA3 and TGF-*β*2 in the third trimester of pregnancy and preeclampsia and on neonatal outcomes.

## 2. Materials and Methods

### 2.1. Objective

52 cases of preeclampsia pregnant women who gave birth in Tengzhou Maternity and Child Health Hospital from June 2020 to December 2020 were selected, including 28 cases of preeclampsia and 24 cases of severe preeclampsia. At the same time, 50 pregnant women with normal delivery during this period were selected as the control group. The selected targets were diagnosed and grouped according to the criteria for preeclampsia in the ninth edition of “Obstetrics and Gynecology.” At the same time, the following conditions are met: (1) singleton live birth, aged 18–40 years old; (2) on-time production inspection, complete the required information; and (3) pregnant women are aware of the study and sign a voluntary consent form. Exclusion criteria are as follows: (1) the enrolled pregnant women have a history of long-term drinking, smoking, or taking drugs during pregnancy; (2) complicated with other serious complications or complications during pregnancy. This study has been approved by the ethics committee of our hospital.

### 2.2. Methods

The age, blood pressure, verified gestational age, gestation times, BMI, weight gain during pregnancy, liver and kidney function test results, and birth weight of newborns were collected. The cord blood S/D ratio was measured within 3 days before delivery. Take 4 ml of the patient's venous blood, leave it at 4°C overnight, centrifuge at 1000 *r*/min for 20 min, extract the serum, put it into a microcentrifuge tube, and place it in a refrigerator at −80°C for later use. The content of HtrA3 and TGF-*β*2 in serum was detected by ELISA (testing reagents were purchased from Shanghai Hailian Biological Co., Ltd.). After the placenta is peeled off, try to avoid calcification, infarction, and vascular areas, cut out the full-thickness placental tissue about 2.0 cm × 2.0 cm × 2.0 cm at a distance of 2 cm from the root of the umbilical cord, rinse it with 0.9% sodium chloride injection, and remove it from the body The specimens were fixed in 10% paraformaldehyde solution for 72 hours within 20 minutes, and the sections were embedded in conventional paraffin, and the average optical density of HtrA3 and TGF-*β*2 in the placenta tissue was calculated by the immunohistochemical staining method combined with ImageJ 180 image processing software (HtrA3 detection reagent purchased from Beijing Boaosen Biotechnology Co., Ltd. TGF-*β*2 is detected with sigma reagent).

### 2.3. Statistics

The statistical analysis software is SPSS 26, and the measurement data are expressed as mean ± standard deviation ($\bar{x}\pm s$). Normally distributed data are compared through single-factor analysis of variance and postmultiple test procedures; the rank sum test method is selected for nonnormal statistical analysis of distribution data. Single correlation data use Pearson linear correlation analysis to determine the correlation between variables. The *r* value not only indicates the correlation but also reflects the direction of the correlation. *P* value <0.05 means that there is statistical significance between the two.

## 3. Results

### 3.1. General Information Comparison

There was no significant difference in the data of the verified gestational age, age, gestation period, and weight gain during pregnancy of the three groups of patients (*P* > 0.05). Before pregnancy, BMI, creatinine, urea nitrogen, and ALT were compared between the control group and the observation group, and the difference in data was statistically significant (*P* < 0.05). The above data of the preeclampsia group was compared with the severe preeclampsia group, and there was no statistical significance among the groups (*P* > 0.05). Pairwise comparisons of systolic blood pressure, diastolic blood pressure, S/D ratio, and newborn birth weight among the three groups showed significant differences (*P* < 0.05) (Table 1).

### 3.2. Comparison of HtrA3 and TGF-*β*2 Expression Levels in Maternal Serum and Placental Tissue

Comparing the contents of HtrA3 and TGF-*β*2 in maternal serum and the average optical density of placental tissue by immunohistochemical staining among the three groups, the results showed that the content of severe preeclampsia was the highest, followed by preeclampsia, and the control group had the lowest content. All are statistically significant (*P* < 0.05).  Table 2 provides the specific values.

### 3.3. Immunohistochemical Color Development in the Placenta of HtrA3 and TGF-*β*2

HtrA3 and TGF-*β*2 show different levels of color in the placenta tissue of pregnant women after enzyme staining. HtrA3 mainly develops color in placental syncytiotrophoblast cells and extravillous trophoblast cells, most of which are located in the cytoplasm. The number of HtrA3-positive staining in the placenta of patients with severe preeclampsia is more than that of preeclampsia, and the staining is deeper, and both of them are more than the number of positive cells in the placenta of normal pregnant women, and the staining is deeper. The expression site of TGF-*β*2 in the placenta is in trophoblast cells, especially in the extracellular matrix of extravillous trophoblast cells. Severe preeclampsia has the darkest staining, followed by preeclampsia, and the placenta of normal pregnant women is relatively lightest (Figures 1 and 2).

### 3.4. Correlation Analysis of HtrA3, TGF-*β*2, and Clinical Data

The correlation value of HtrA3 in maternal serum and placenta tissue and newborn birth weight was (*r* = −0.508, −0.64), which was negatively correlated; the correlation value of HtrA3 with umbilical artery S/D was (*r* = 0.565, 0.473), respectively. It is positively correlated. The correlation value between TGF-*β*2 and newborn birth weight was (*r* = −0.478, −0.539), which was negatively correlated; the correlation value of TGF-*β*2 with umbilical artery S/D was (*r* = 0.453, 0.492), which was positively correlated. The *P* values were all <0.05, and the difference between pairwise was statistically significant, as given in Table 3.

## 4. Discussion

### 4.1. Overview of Preeclampsia

Experts consider the preeclampsia to be a placenta-derived disease. Due to its complex pathological process and diverse clinical manifestations, its specific pathogenesis has not yet been fully ascertained. Both the classic “two-stage theory” and the refined “six-stage model” point out that trophoblast cells are insufficiently differentiated, migrated, and invaded, preventing them from invading into the myometrium, resulting in obstructed and changed uterine spiral artery remodeling. In the local microenvironment, a variety of humoral factors are abnormally expressed, which ultimately results in the dysfunction of multiple organs in pregnant women and a series of clinical manifestations. This process is recognized as one of the mechanisms of preeclampsia [5].

### 4.2. The Relationship between HtrA3 and Preeclampsia

HtrA3 is a serine protease associated with pregnancy. There are two subtypes of long and short (i.e., HtrA3-1 and HtrA3-s). HtrA3 is mainly expressed in decidual cells, syncytial trophoblast cells, and extravillous trophoblast cells during pregnancy. It can degrade the extracellular matrix, regulate the microenvironment of decidual cells, and inhibit the proliferation, differentiation, and invasion of trophoblasts, thereby affecting placental development [6]. Studies have found that HtrA3 is most produced in the first 3 months of pregnancy, and the abnormal increase in serum HtrA3 at 13-14 weeks of gestation is related to preeclampsia. Yee et al. detected serum HtrA3 levels at 15 and 20 weeks of gestation, respectively. The control found that pregnant women with late-onset preeclampsia or small-for-gestational-age infants had a significant reduction in serum HtrA3 levels at 15 weeks of gestation. The 15-week reduction in HtrA3 levels can be used to early predict the birth of late-onset preeclampsia and small-for-gestational-age infants and provide a basis for intervention and early treatment [7]. Wang et al. used two highly specific monoclonal antibodies to detect HtrA3 in the serum of pregnant women at 11–13 weeks of pregnancy and found that the level of HtrA3-1 was significantly increased in patients with late-onset preeclampsia, while in patients with early onset preeclampsia. The ratio of HtrA3-l/HtrA3-s is significantly lower. These data confirm the potential use of HtrA3 in the early detection of preeclampsia [8]. In this study, the maternal serum and placental tissues of the third trimester of pregnancy were tested in different ways. It was found that the levels of HtrA3 in the maternal serum and placental tissues of severe preeclampsia and preeclampsia were higher than those in the control group. Based on this, it is speculated that abnormal expression of HtrA3 is associated with eclampsia. Preeclampsia is related, and the severity of preeclampsia can be inferred based on the content of HtrA3.

### 4.3. The Relationship between TGF-*β*2 and Preeclampsia

Transforming growth factor (TGF-*β*) can control the proliferation, differentiation, and invasion of trophoblast cells through negative regulation during pregnancy. Foreign scholars like Prossler et al. established an EVT invasion model in early pregnancy to increase the concentration of exogenous TGF-*β*2 and used high-throughput quantitative methods to detect that the invasion range of EVT gradually decreased with the increase of TGF-*β*2 concentration, thus proving that TGF -*β*2 can inhibit EVT invasion in early pregnancy [7, 9]. Domestic scholars such as Li et al. used reverse transcription-polymerase chain reaction and Western blotting to detect the expression of TGF-*β*2 mRNA and the protein content in the placenta and found that the ROD value in the preeclampsia group was higher than that in the normal pregnancy group [9]. The level of its value is closely related to several clinical indications that symbolize the severity of the disease.

### 4.4. The Relationship between the Expression of HtrA3 and TGF-*β*2 in Maternal Serum and Placenta Tissue and Clinical Indicators

The S/D value of umbilical blood flow is a sensitive indicator that reflects the fetal circulatory perfusion of the placenta. As the gestational age increases, the S/D ratio will decrease [10]. In patients with preeclampsia, the placenta accreta becomes shallow, the circulatory resistance increases, and the S/D value increases. Nagar and other studies have shown that abnormally elevated S/D also has a predictive value for adverse pregnancy outcomes such as intrauterine growth restriction and preeclampsia [11]. HtrA3 and TGF-*β*2 are related to the increase of the S/D value, which is helpful for the early diagnosis of preeclampsia and small-for-gestational-age infants, and can affect the birthweight of newborns and may even affect the distribution and content of body fat in the future [12–14]. The correlation analysis of the data using Pearson straight line in this study also confirmed the correlation between the expression levels of HtrA3 and TGF-*β*2 and the S/D ratio, that is, positively correlated and negatively correlated with the birthweight of the newborn.

## 5. Conclusion

In summary, the abnormally high expression of HtrA3 and TGF-*β*2 is correlated with preeclampsia and related clinical indicators. However, because this study is a small sample data study, the practical value of the experimental results in the clinical work requires a large number of samples. The information is further confirmed.

## Figures and Tables

**Figure 1:** Expressions of HtrA3 in the placenta of normal pregnancy, PE, and severe PE (×200). (a) Normal pregnancy. (b) PE. (c) Severe PE.

**Figure 2:** Expressions of TGF-*β*2 in the placenta of normal pregnancy, PE, and severe PE (×200). (a) Normal pregnancy. (b) PE. (c) Severe PE.

**Table 1:** General data of comparison of research objects.

Project	Control group	Preeclampsia group	Severe preeclampsia group
Gestational week	38.88 ± 0.19	38.64 ± 0.13	38.37 ± 0.27
Age	29.54 ± 5.44	28.61 ± 6.02	29.67 ± 6.61
Pregnancy times	2.62 ± 1.32	2.57 ± 1.26	2.25 ± 0.98
Weight gain	16.02 ± 6.06	14.61 ± 6.53	14.42 ± 5.16
BMI	23.28 ± 3.86	25.66 ± 5.24	26.22 ± 3.82^&^
Systolic blood pressure	117.68 ± 10.38	143.50 ± 11.75^@#^	163.33 ± 12.36^&^
Diastolic blood pressure	75.34 ± 8.42	95.75 ± 10.98^@#^	106.38 ± 7.54^&^
S/D	2.02 ± 0.27	2.20 ± 0.30^@#^	2.57 ± 0.31^&^
Newborn weight	3506.00 ± 454.18	3118 ± 387.23^@#^	2845.8 ± 461.01^&^
Amniotic fluid pollution	6%	17.85%^@#^	76.15%^&^
Creatinine	48.22 ± 6.87	54.21 ± 12.27^@^	57.42 ± 12.84^&^
Urea nitrogen	2.71 ± 1.58	3.62 ± 2.18^@^	3.67 ± 1.18^&^
ALT	9.82 ± 4.63	13.02 ± 8.07^@^	21.14 ± 28.62^&^
AST	15.05 ± 3.37	18.61 ± 13.41^@^	24.88 ± 23.25^&^

^@^ *P* < 0.05, preeclampsia vs. the control group. ^#^*P* < 0.05, severe preeclampsia vs. preeclampsia. ^&^*P* < 0.05, severe preeclampsia vs. the control group.

**Table 2:** Comparison of HtrA3 and TGF-*β*2 expression levels in maternal serum and placenta tissue.

Group	HTRA3		TGF-*β*2	
	Maternal serum	Placental tissue	Maternal serum	Placental tissue
Control group	532.80 ± 325.10	0.423 ± 0.238	624.54 ± 284.05	0.418 ± 0.179
Preeclampsia	873.29 ± 469.45^@#^	0.44 ± 0.121^@#^	874.96 ± 327.31^@#^	0.42 ± 0.127^@#^
Severe preeclampsia	1484.13 ± 510.61^&^	0.464 ± 0.303^&^	1273.00 ± 475.28^&^	0.449 ± 0.314^&^

^@^ *P* < 0.05, preeclampsia vs. the control group. ^#^*P* < 0.05, severe preeclampsia vs. preeclampsia. ^&^*P* < 0.05, severe preeclampsia vs. the control group.

**Table 3:** Correlation of HtrA3 and TGF-*β*2 in maternal serum and placental tissue with newborn weight and S/D ratio.

	HTRA3				TGF-*β*2			
	Maternal serum		Placental tissue		Maternal serum		Placental tissue	
	*r*	*P*	*r*	*P*	*r*	*P*	*r*	*P*
S/D	0.565	<0.05	0.473	<0.05	0.453	<0.05	0.492	<0.05
Newborn birth weight	−0.508	<0.05	−0.64	<0.05	−0.478	<0.05	−0.539	<0.05

## Data Availability

The datasets used and/or analyzed during the current study are available from the corresponding author upon request.
